RETRACTED

# Research on the Dilemma and Path of Rural Industry Integration and Internet Revitalization Driven by e-Commerce

**DOI:** 10.1155/2022/8665698

**Published:** 2022-09-13

**Authors:** Feng Xu

**Affiliations:** Yiwu Industrial & Commercial College, Yiwu 322000, China

## Abstract

Because e-commerce is based on the Internet, it has the advantages of fast response speed and strong promotion ability, which potentially mitigates the problems of low popularity and unreasonable industrial structure in the development of rural industries. This paper integrates Internet technology, studies in detail the functional process of rural industries integrating the Internet, and establishes the corresponding platform. Then, it analyzes the problems of rural industrial integration of the Internet to achieve rural revitalization and applies this rural industrial integration of the Internet revitalization platform to the rural development of different cities. By studying the difficulties in rural industry among cities, this paper compares and analyzes the optimization measures of this path and puts forward the corresponding solutions. In short, this paper integrates rural industry with Internet technology, which greatly improves the popularity of rural industry, optimizes the rural industrial structure, and provides ideas and experimental support for the realization of rural revitalization.

## 1. Introduction

With the sustainable development of the agricultural economy, China's grain output has increased steadily, and farmers' income has also increased significantly. Nowadays, with the continuous optimization of China's economic structure, the consumption demand of urban and rural residents has changed qualitatively [1]. In addition, farmers are also developing in the direction of urbanization. Most of them go out to work and few people grow agricultural crops. Accordingly, the relationship between agricultural supply and demand has gradually changed from “production-oriented” to “consumption-oriented.” In this context, problems such as the gradual marginalization of farmers' status, the rising cost of agricultural production, the unreasonable allocation of rural resource elements, and the continuous deterioration of the ecological environment are emerging one after another. Adhering to the traditional mode of agricultural industrialization has been unsustainable, and there is an urgent need to build a new development mode and actively promote the integrated development of rural industries [2].

Rural industrial integration refers to the mutual penetration, integration, and common development of primary, secondary, and tertiary industries such as agriculture, industry, service industry, and information industry at different structural levels in rural areas in the same industry, industrial, chain and industrial network, with the high-end dominating the low-end, the advanced driving the backward, and the vertical radiation horizontal so that the low-end industry becomes a part of the high-end industry, the knowledge operation growth mode, and rural industrial management mode to complete the overall transformation and upgrading of the industry [3]. The integration of rural industries can not only broaden the development space of rural industries, optimize the rural industrial structure, and form new forms of rural industries but also help farmers increase their income and become rich and narrow the development gap between urban and rural areas.

RETRACTED

In the process of rural industrial integration development, we have experienced the following development background [4, 5]. First of all, the main bodies of the production, processing, sales, and other links of agricultural products are independent, and there is no interest division relationship between them. Coupled with the lack of environmental protection awareness, they do not pay attention to protecting the environment in production and operation, plunder agricultural resources wantonly, and discharge high polluting substances and harmful gases excessively, which leads to the unreasonable allocation of agricultural production factors, and the former “green mountains and green waters” are gradually disappearing. At present, agriculture is in a weak position, the agricultural economic benefits are always low, the growth of farmers' economic income is still weak, and the rural ecological environment continues to deteriorate. We must seek a way out, actively build the interest connection mechanism of agricultural business entities and economic entities, and provide guarantee for promoting the integrated development of rural industries.

Second, compared with other industries, the economic benefits brought by agriculture to workers are relatively low, resulting in rural decline, population aging, and other problems. To reverse this situation, we must actively promote the integrated development of rural industries, make great efforts to extend the industrial chain, and realize the value-added of agricultural production [6].

Third, to improve the overall efficiency of agricultural production, China began to actively explore the development mode of agricultural industry as early as the 1990s. However, with this development model, farmers play a limited role in the whole business industrial chain, and can only provide agricultural raw materials for leading enterprises from the source [7]. However, farmers do not participate in the subsequent processing, transportation, sales, and other links of enterprises, so the benefits that farmers can share are only limited to the supply of agricultural products.

RETRACTED

Finally, today, with the acceleration of the process of urban–rural integration, earth-shaking changes have taken place in both people's lifestyle and consumer demand and structure. On the one hand, urban and rural residents continue to pay more attention to dietary structure, food safety, and health preservation, and their consumption demand for agricultural products is not satisfied with solving the problem of food and clothing. Quality and safety have become hard indicators for consumers to buy agricultural products. With the substantial improvement of residents' income level, personalization and high end of agricultural products have also begun to become the focus of many consumers [8]. On the other hand, the demand of urban and rural residents for rural resources has changed from simplification to diversification. To meet the needs of consumers and adapt to the changes in the relationship between supply and demand as soon as possible, we must promote the close integration of agriculture, processing industry, and service industry [9].

At present, in the process of rural industrial integration development, the overall level of agricultural industrialization in China is not high, the brand influence is small, and the industrial integration system is not perfect, which seriously restricts the development of rural industrial integration. There are the following problems [10, 11]:

(1) The implementation of rural industrial integration policy is not in place. At present, China has issued a series of policies to support the integrated development of rural industries. However, due to the short development time of industrial integration in most rural areas of China, there is no mature development system, and the development experience and methods are still in the exploratory stage. It is difficult for local government departments and enterprises to match the application of policies with development issues, resulting in the implementation of relevant policies not in place.

(2) The homogenization of rural industrial integration is serious. At present, the homogenization of rural industrial integration in China is serious. To pursue short-term interests, some rural areas blindly follow the trend of the market and ignore their own developmental advantages and local characteristic resources, which leads to the lack of distinctive features of products and vicious competition with other regions, which is not conducive to the long-term development of rural economy.

(3) The main force of rural industrial integration is missing. The integrated development of rural industries is not only an opportunity for rural economic development but also contains many risks. Many rural industrial entities are afraid of crossing the river, unwilling to bear the risks of integrated development, timid, and adopt an overly conservative industrial development mode, which is difficult to form a strong development force.

(4) Lack of perfect rural industrial integration service mechanism. Promoting the integrated development of rural industries is inseparable from the corresponding information, technology, and service support. However, most rural areas in China have not established a perfect rural industrial integration service mechanism. The services that can be provided to the main body of rural industrial integration are only limited to the supply of means of production, production technology, and marketing means. The service efficiency is low and the quality is poor, which is difficult to promote the development of rural industrial integration.

RETRACTED

The emergence of network technology has promoted the birth of the Internet, and the development of the Internet has not only changed our lives but also promoted the reconstruction of business models, among which the most far-reaching impact is the development of e-commerce economy [12]. However, the market penetration of e-commerce of agricultural products is still low, and the problems of poor consumption experience and high logistics costs have become important factors restricting the development of traditional e-commerce of agricultural products. With the continuous upgrading of consumer demand, e-commerce of agricultural products must also continue to innovate to meet the personalized needs of consumers [13, 14].

Electronic commerce refers to a series of business activities carried out with the support of computer Internet. It not only includes all important links in traditional trade but also innovates the traditional trade mode, which fully reflects the advantages of e-commerce in the form of low cost and high efficiency. e-Commerce can increase the competitive advantage of enterprises, improve the management level of enterprises, and help enterprises obtain more market information, which is of great significance [15]. Its effect on enterprises is long-term and strategic, so the economic benefits of investment are difficult to see in the short term. Domestic enterprises should fully understand the cost and ultimate advantages of e-commerce, and avoid losing the opportunity for enterprise development to obtain short-term benefits.

e-Commerce can promote rural products to the Internet through Internet technology, so that customers can understand rural products, and then promote the marketing of rural products through online live broadcasting, so as to promote the development of rural industries.

e-Commerce has the following advantages [16, 17]. First, e-commerce has the advantages of low cost, fast speed, and high efficiency. The e-commerce model mainly relies on the Internet to build a worldwide marketing network, reducing the intermediate links of traditional trade, thus greatly saving the cost of management and personnel links. Second, e-commerce has high quality and a large market. e-Commerce can reduce the obstacles of space and realize cross-regional and cross-border transactions. In addition to ensuring that the transactions of original customers are completed according to quality and quantity, it can also open up potential hidden customers and expand the market through online advertising. Third, e-commerce has the advantage of improving the competitiveness of enterprises [18]. The traditional way of trade makes the management mode of enterprises pyramid-like, top-down control management. In the e-commerce environment, the internal information exchange of enterprises is no longer confined to the original “level-by-level transmission” or “one-to-one transmission” mode, but realizes the flexible mainstream mode of “one to many” or “many to many,” forming an efficient management and business process.

RETRACTED

Demand is an important factor driving the development of e-commerce for agricultural products. With the upgrading of consumer demand, e-commerce for agricultural products is also in dynamic development to meet changing needs. From the perspective of economics, demand, on the one hand, is expressed as a preference for goods [19, 20]. On the other hand, it is expressed as the ability to pay. In terms of preferences, consumers' demand for agricultural products has shifted from focusing on quantity and variety to focus on quality and life, and their requirements for quality, freshness, safety, brand, added value, purchase convenience, and rapidity are becoming higher and higher [21]. In terms of payment ability, with the rapid development of economy, China's residents' income level continues to improve, consumers have a certain ability to pay for high-quality and brand agricultural products, and consumers' purchase of agricultural products has changed from “can buy” to “selective purchase.” In the Internet era, consumer behavior has changed significantly, and the change in consumption mode will promote the continuous reform and innovation of agricultural e-commerce [22].

Based on Internet technology, Chen [23] discusses the problems of rural industrial integration development and puts forward measures to promote rural industrial economy, which is of great significance. Yang and Saearani [24] study the development of Internet integration in rural industries driven by e-commerce. By optimizing the hierarchical structure between e-commerce and rural industries, e-commerce can promote rural revitalization. Based on the rural revitalization strategy, Hong [25] studied the integration of rural industries and proposed that we must develop new forms of rural industries, so as to promote the mutual penetration and common development of rural industries at different levels. Chen [26] reconstructs the development of rural industry driven by e-commerce by studying the diversification of e-commerce, combined with the development needs and operation mode of rural industry, which has a good reference value for the realization of rural revitalization at present.

RETRACTED

Based on this, driven by e-commerce, to realize the National Rural Revitalization Strategy, this paper establishes the corresponding model analysis according to the current development status of rural industry and the integration of Internet technology. Then, it studies the problems and difficulties of rural industry integration and Internet revitalization driven by e-commerce between different cities and puts forward the corresponding solutions. In general, this paper provides some experimental and theoretical support for the development of rural industry and the realization of rural revitalization, and has good reference significance.

## 2. Analysis of Internet Model of Rural Industrial Integration

### 2.1. Internet Function Principle of Rural Industrial Integration

Driven by e-commerce, the integration of rural industries into the Internet requires a corresponding industrial division of labor. If the rural industry can solve the problem alone, then those who solve this problem can have corresponding experience, and they can better solve similar problems. However, if the rural industry is combined with industries in other fields, the final results will be divided, and almost all other types of rural industries will face similar problems. For the Internet, it is the best decision to choose the least resources to solve the problem and strengthen the cooperation effect to maximize the innovation results. The effective function can reduce the interference of invalid factors, which can describe and solve the problem in detail, and has the optimal solution. Therefore, in the environment of e-commerce, the utility function method is proposed to be used in the research of rural industrial integration Internet.

RETRACTED

It is the best decision for any rural industry to choose the least Internet resources to achieve rural revitalization so that the development of rural industrial economy can be maximized, and it is also the best way to choose the ideal rural industry. Therefore, we can express it with the following equation:

(1) $$\begin{array}{c} \mu_{i}=\frac{1}{\left|C_{i}\right|}+\underset{j\neq isti\in C_{i}}{\sum }\frac{1}{\left|C_{i}\right|}, \end{array}$$

where *C_i_* refers to the number of rural industries, *μ_i_* indicates the function of the Internet, which has the functions of rapidity, accuracy, and universality. In the coordination network, if rural industries want to integrate with the Internet, they should adopt the following methods to choose.

Suppose *C* = {*C*_1_, *C*_2_, ⋯, *C*_*N*_}, where *C_N_* represents the number of the *N*-th industry in the rural industry. *A* = {*a*_1_, *a*_2_, ⋯, *a*_*i*_} represents the working efficiency of this Internet technology. Because rural industries need the Internet to upgrade and develop, the higher the efficiency of the Internet, the easier it is for rural industries to develop, so the correlation between rural industry and the Internet can be obtained from the following equation:

(2) $$\begin{array}{c} A_{j}=\left\{a_{j1},a_{j2},\cdots ,a_{ji}\right\},j=1,2,\cdots ,n,0<a_{ji}<1. \end{array}$$

The weighted method can process the data finely and screen out the invalid data, which can improve the accuracy of the data and reduce the error. Therefore, comprehensively evaluate and optimize the rural industry, select the weighting method, set the weighting factor according to the Internet technology, and conduct quantitative calculation. The evaluation results are as follows:

(3) $$\begin{array}{c} \beta_{i}=1-\overset{5}{\underset{i=1}{\sum }}C_{i}\left|a_{ji}-b_{i}\right|,i=1,2,\cdots ,n;j=1,2,3,4,5, \end{array}$$

(4) $$\begin{array}{c} \overset{5}{\underset{i=1}{\sum }}c_{i}=1,i=1,2,3,4,5. \end{array}$$

Where *β_i_* represents the data of rural industrial optimization. According to the above methods, through the comprehensive analysis of the operation mode and future development of the rural industry through Internet technology, we can get the integration degree of rural industry and Internet technology and, finally, realize the rural revitalization of rural areas.

### 2.2. Model of Rural Industrial Integration and Internet Revitalization

Because e-commerce is based on the Internet and the development of rural industries needs e-commerce promotion, so as to obtain good benefits. In the context of e-commerce driven, the probability of integration of rural industry and Internet technology is *x* and *y*, respectively, and the probability of noncooperation is 1 – *x* and 1 – *y*, respectively. Then, the expected benefits of e-commerce platforms adopting the cooperation strategy to implement innovation are:

(5) $$\begin{array}{c} \underset{\text{ec}}{\prod }=y\left(\pi_{\text{e}}+∆\pi_{\text{e}}-C_{\text{oe}}\right)+\left(1-y\right)\left(\pi_{\text{e}}-C_{\text{oe}}-C_{\text{e}}\right). \end{array}$$

The expected benefits of e-commerce platforms adopting the noncooperative strategy to implement innovation are:

(6) $$\begin{array}{c} \underset{\text{enc}}{\prod }=y\left(\pi_{\text{e}}+B_{\text{e}}\right)+\left(1-y\right)\pi_{\text{e}}. \end{array}$$

The average expected return of e-commerce platform innovation is:

(7) $$\begin{array}{c} \underset{\text{e}}{\prod }=x\underset{\text{ec}}{\prod }+\underset{\text{enc}}{\prod }\left(1-x\right). \end{array}$$

Therefore, the replication dynamic equation of e-commerce platforms is:

(8) $$\begin{array}{c} \frac{\text{d}x}{\text{d}t}=x\left(1-x\right)\left[y\left(∆\pi_{\text{e}}-B_{\text{e}}+C_{\text{e}}\right)-\left(C_{\text{oe}}+C_{\text{e}}\right)\right]. \end{array}$$

It is worth noting that optimizing the Internet improves its popularity, strengthens its publicity, and upgrades rural industries.

RETRACTED

The replication dynamic equation during fusion is:

(9) $$\begin{array}{c} \frac{\text{d}y}{\text{d}t}=y\left(1-y\right)\left[x\left(∆\pi_{\text{h}}-B_{\text{h}}+C_{\text{h}}\right)-\left(C_{\text{oh}}+C_{\text{h}}\right)\right]. \end{array}$$

Because the Jacobian matrix has the advantage of rapid response, which can accurately screen the cooperation behavior between e-commerce platform and entity business, and has the advantage of convenience and simplicity. Therefore, the local stability analysis method of Jacobian matrix can be used, and we can get that the cooperation behavior between e-commerce platform and entity business is an equilibrium point with five coordination relations: point *A* (0, 1), point *B* (1, 1), point *C* (1, 0), point *O* (0, 0), and point *D* (*x_D_*,*y_D_*), and the equation is as follows:

(10) $$\begin{array}{c} x_{D}=\frac{C_{\text{h}}+C_{\text{oh}}}{∆\pi_{\text{h}}-B_{\text{h}}+C_{\text{h}}},\;y_{D}=\frac{C_{\text{oe}}+C_{\text{e}}}{∆\pi_{\text{e}}-B_{\text{e}}+C_{\text{e}}}. \end{array}$$

Through verification, points *A*, *B*, *C*, *D*, and *O* are the five equilibrium points of the system, and point *B* (1, 1) or point *O* (0, 0) is the evolutionary stability point, where point *B* (1, 1) is the evolutionary stability point where both parties adopt cooperative strategies, and point *O* (0, 0) is the evolutionary stability point where both parties adopt betrayal strategies or noncooperation. Furthermore, by improving the precise position of the data points, the Jacobian matrix is used to optimize them, so as to ensure the stability of the evolutionary stability point. In addition, points *C* (1, 0) and *A* (0, 1) are the unstable points of the system, and point *D* (*x_D_*, *y_D_*) is the saddle point.

RETRACTED

### 2.3. Construction of Internet Platform for Rural Industrial Integration Driven by e-Commerce

In the development of e-commerce, it needs to be combined with rural industries, which is also closely related to Internet technology. However, in the operation of e-commerce, it is necessary to conduct in-depth and detailed innovation management at each stage of the business model innovation process to ensure that the impact of the uncertainty of the innovation process on the innovation results is minimized so that the business model can achieve the innovation goals according to the established plan, as shown in Figure 1.

Rural industries need to carry out e-business model innovation under the Internet according to their own conditions and innovation capabilities. The ability of innovation path selection and strategy formulation is insufficient, and it will not be able to make the right direction for e-commerce model innovation. Lack of innovation organization capacity will not provide team guarantee and planned arrangement support for rural industrial model innovation. If the design ability and implementation ability are insufficient, the mode design and implementation of the new mode will not be completed. Through the construction and evaluation of the innovation ability index system, the evaluation management of the innovation ability of rural industrial e-commerce model can timely point out the lack of innovation ability of the whole or all parts of the rural industry, and then quickly adjust to avoid the delay or lower than expected effect of rural industrial e-commerce innovation caused by the lack of innovation ability. Therefore, the Internet platform for rural industry integration driven by e-commerce is extremely important for the development mode of rural industry, to better realize the rural revitalization strategy. The specific platform diagram is shown in Figure 2. It is worth noting that during the construction of the platform, we fully investigated the integration of rural industries and the Internet between different cities across the country, and carried out optimization analysis on this basis, to ensure the wide applicability of the platform.

## 3. Research on Rural Industrial Integration and Internet Revitalization between Different Cities Driven by e-Commerce

### 3.1. Dilemma Analysis of Rural Industry Integration and Internet Revitalization between Different Cities Driven by e-Commerce

As we all know, the distribution of rural population is relatively scattered and far away. This inherent form greatly affects the downward accessibility of e-commerce, and it is difficult to form the agglomeration effect of e-commerce consumption in urban communities. The production and marketing strategy of rural live broadcast e-commerce has a typical “export-oriented” feature, that is, the rural origin is not the home of consumption, but up to the city. Therefore, the main way for rural live broadcast e-commerce to drive local economic growth is to rely on supply chain and logistics distribution. Although the popularity of the Internet and the application of digital technology can reduce the “information gap,” for the modernization of space governance, the difficulties still focus on the “last mile” of e-commerce logistics distribution, and the delivery efficiency of agricultural products into cities, especially fresh agricultural products, and the cold chain guarantee system are relatively lagging behind. At the same time, there are obvious differences in the development level of rural e-commerce in different regions, and the industrial foundation is also divided into strong and weak. For villages with weak e-commerce foundation and small scale, there is great upward pressure on agricultural products. The goal of the rural revitalization strategy is not only to increase agricultural output and enrich farmers but also to improve the overall appearance of rural production and life, and create new market opportunities through new business forms. The capture of this opportunity needs to be based on building and consolidating industries, especially traditional and advantageous industries, to create rural dividends of the new model of e-commerce.

RETRACTED

Figure 3 shows the development of Internet platform for rural industrial integration between different cities driven by e-commerce. It can be seen from this that driven by e-commerce, the development of Internet platforms for rural industrial integration between different cities shows a gradual and slow downward trend with the increase over time. The development of Shanghai and Beijing is better, both reaching more than 65%, and the initial development of Shanghai is the highest, and then decreased, while the development of Beijing presents a relatively stable development trend. The development of the Internet platform for rural industrial integration in Chongqing ranks third and Tianjin ranks last. The development of these two cities shows a similar law of change over time, both of which are first reduced and then increased and tend to be stable. The main factor causing the difference in the development of the Internet platform for rural industrial integration between the above different cities is the difference in economic capacity, scientific, and technological cultural levels among the four cities. Among them, development in Beijing and Shanghai, as China's strong cities in science, technology, culture, and economic level, must be in the top two. The economic and technological level of Chongqing is higher than that of Tianjin, so it ranks third and Tianjin ranks fourth. In general, to better promote the development of rural industrial integration Internet between different cities, we should train and educate local farmers to improve their enthusiasm. At the same time, publicize the Internet accordingly, and realistically focus on the comprehensive development of key points according to the economic and cultural status of different cities, and finally, achieve the goal of rural revitalization.

### 3.2. The Ability of Rural Industry Integration and Internet Revitalization between Different Cities Driven by e-Commerce

Affected by the traditional agricultural and rural development model, most rural left behind people are still attached to the “small-scale peasant economy,” satisfied with self-sufficient farming life, and lack the awareness of active participation in digital villages and rural live broadcasting. With the development of the Internet, live broadcasting and delivery have developed rapidly. However, with the rapid development of live broadcasting, we should also see some problems in its business model innovation, among which the professional quality and ability of live-broadcasting personnel are the key. Due to the influence of the star effect of some so-called ”top celebrities” in live broadcasting, it is easy for entrepreneurs to underestimate or misjudge the difficulty of the development of the new model of live-broadcasting e-commerce. From the perspective of the industrial cycle stage, this is particularly important for the initial development of rural live-broadcasting e-commerce. In terms of structure, due to the single rural industry, backward transportation, slow economic development, and insufficient publicity for rural areas, it is unable to provide a good development space for young and middle-aged people, which has caused the outflow of rural talents. Meanwhile, the main participants of live broadcast e-commerce sinking villages are still rich experts, Xinxiang sages, and returning youth. In some areas, there are structural problems such as “hollow villages,” old and weak left behind personnel, and low willingness of young workers to revitalize the village economy. There is a lack of professional direct broadcast e-commerce leaders in rural areas, which has not yet formed a strong village-level driving effect. In terms of innovation, there are simple models to copy, and the depth of imitation learning is not enough so that the professional ability to carry out marketing activities with the help of e-commerce or short video platforms is insufficient, the dependence on rural collectives and entrepreneurial leaders is strong, the spontaneous motivation is insufficient, and the professional and innovative capacity-building of live-broadcasting needs to be enhanced.

RETRACTED

Figure 4 shows the proportion rate of rural industry integration and Internet revitalization among different cities driven by e-commerce. It can be seen that Beijing and Shanghai pay more attention to innovation and learning ability, and the proportion of urban quality and structure is relatively close. The learning ability of Chongqing is better, and the urban quality of Tianjin is better, but the innovation ability of these two cities is slightly insufficient, which leads to some problems in the integration of rural industries in the two cities and the Internet, which is not conducive to the realization of rural revitalization. The innovation ability of cities is crucial to the development of rural industries, and it is also a key issue to promote rural revitalization. Therefore, while trying to balance the problems of innovation, learning, quality, and structure between different cities, we should also pay attention to the cultivation of innovation ability. After all, innovation ability is a continuous driving force for the development of a city. Only in this way can we put forward corresponding optimization measures according to the dilemma of the integration of rural industries with the Internet, so as to promote the all-round development of rural industries and realize the strategy of rural revitalization.

### 3.3. Talent Demand of Rural Industry Integration and Internet Revitalization between Different Cities Driven by e-Commerce

e-Commerce entering villages and villages is an important way to boost the development of agricultural and rural modernization, and it is also a new engine to comprehensively promote rural revitalization. However, with the rapid development of rural e-commerce, it still faces challenges such as the structural imbalance of human capital, which hinders the effective rooting of new e-commerce formats and models in the practice of rural revitalization. In particular, there is a large gap of talents who love agriculture and are good at management, and know technology so that rural e-commerce is easy to fall into the dilemma of weak sustainability after initial growth, affecting the effect of rural revitalization. Human capital is the core element of rural revitalization, and talents are the first resource for live e-commerce to help rural revitalization. From the perspective of the supply of social resources, on the one hand, various talent projects at all levels “build nests and attract Phoenix,” promoting the introduction of talents to take root in the countryside. On the other hand, identify and cultivate rural local talents in a multichannel and all-round way, and strive to build a live broadcast e-commerce “local leader/leader” committed to the cause of rural revitalization, giving play to the radiation effect from the point to the area. Either relying on the existing platform or taking live e-commerce as the educational theme, build a special training institution for rural revitalization talents, take the opportunity of rural revitalization, implement the local live e-commerce talent training plan, create a village level “e-commerce live room,” establish a town level rural revitalization lecture hall, and form a demand-driven “single-point” online and offline knowledge transmission mode.

RETRACTED

Figure 5 shows the educational background of talents in the Internet revitalization of rural industrial integration between different cities driven by e-commerce. It can be seen that the proportion of undergraduates engaged in e-commerce industry in Beijing and Shanghai is the largest, followed by junior college students and master's students, and the proportion of doctoral students is the lowest. Chongqing and Tianjin have the largest proportion of junior college students, followed by undergraduate and master's students, and only a small number of talents have doctoral degrees. The main reason is that Beijing and Shanghai are rich in educational resources, and most highly educated talents will devote themselves to grass-roots construction after graduation, which is conducive to rural revitalization and rural industrial upgrading. However, the educational resources in Chongqing and Tianjin are relatively general, and the training of talents is insufficient, resulting in fewer highly educated talents to participate in the revitalization of rural areas. Therefore, to better realize the rural revitalization strategy, we should strengthen the training of local talents, set up education, and vigorously encourage village students to study hard. At the same time, we should strengthen the publicity of rural policies, introduce highly educated talents, encourage and support highly educated talents to enter the grass-roots level for training, so as to promote the upgrading and rational allocation of rural industries, and improve the happiness index of local farmers.

RETRACTED

### 3.4. Analysis of the Integration Degree of Rural Industry Integration Internet between Different Cities Driven by e-Commerce

The key to rural revitalization is to revitalize industries. With the in-depth promotion of the rural revitalization strategy, problems such as insufficient innovation and rough services in existing industries have seriously hindered agricultural reform. Live broadcast e-commerce is an important starting point for rural revitalization to achieve industrial prosperity and economic growth. It is an effective new type of business to accelerate industrial adjustment and structural upgrading and promote industrial integration. The primary task of live broadcast e-commerce to drive the integration of rural industries is to complete its own transformation and upgrading. The key to the innovative development of rural industries lies in the adjustment of product supply structure. For example, the existing rural e-commerce is upgraded to a digital rural economic format of “e-commerce + live broadcasting.” On the basis of existing or newly built rural industries, we should explore the coincidence of innovative development in terms of interaction and integration. The second is to enlarge the superposition effect of “live e-commerce + digital village,” and promote the industrial characterization and value-added development of rural economy through the shaping of new agricultural brands and the guidance of characteristic demonstration bases. Starting from the rural resource endowment, we should actively explore the “live broadcast +” rural revitalization model. While relying on the live broadcast of rural agricultural and sideline products to bring goods, we should explore the diversified functions of agriculture and extend the value chain. For example, through live broadcast to help agriculture, we can drive the integration of rural culture and tourism, the protection of traditional villages, and other business forms to add value. Finally, the “live + e-commerce” strategy of rural industrial integration must adhere to the guarantee of improving the infrastructure and public service system and realize the reasonable flow and two-way accommodation of urban and rural factors in industrial supporting facilities, platform construction, market expansion, investment, financing services, etc.

Figure 6 shows the fusion degree in the Internet revitalization of rural industrial integration between different cities driven by e-commerce. It can be seen that the integration degree of Beijing and Shanghai is high, both higher than 90%, while the integration degree of Beijing is close to 95%, followed by Chongqing and Tianjin. The main reason for the difference in the integration degree of rural industry and Internet in different cities may be related to the economic development and education of each city. As we all know, Beijing and Shanghai have the best educational resources in the country and the best economic strength, so local rural industries can quickly integrate with the Internet. The economic capacity of Chongqing is better than that of Tianjin, and the educational resources are equivalent, which leads to the higher integration of rural industry and Internet in Chongqing than that in Tianjin. Therefore, to better promote the integration of rural industries and the Internet between different cities, we should develop local economy and education according to local conditions, so as to provide backup resources for rural revitalization and effectively realize the all-round development of rural economy.

RETRACTED

### 3.5. Diversified System Construction of Internet Platform for Rural Industry Integration between Different Cities Driven by e-Commerce

Farmers are the main body of rural construction in China. The improvement of farmers' quality and ability largely determines the overall value and prospects of rural revitalization. Especially in the period of normalization of epidemic prevention and control, how to activate the vitality of the rural bottom through new business forms and new models, and ensure that rural economic development is not “off-line” or “Involution” is the prerequisite task. Considering the diversity of live broadcast e-commerce and the complexity of rural revitalization, the support of social forces is indispensable for rural revitalization through live broadcast e-commerce. First, we should vigorously guide and support local farmers to participate in live e-commerce, and encourage college students and urban migrant workers to return home and start businesses. Second, improving the mechanism of grass-roots leaders' live broadcasting and goods to help rural revitalization is not only the embodiment of helping farmers serve and complete performance appraisal but also the embodiment of keeping close contact with the masses and changing work style, which is more conducive to the formation of a leadership demonstration role. Third, by constantly improving the business environment, encouraging and absorbing the technical support of all kinds of enterprises and social forces, we should adopt a variety of co-construction and sharing methods to seize opportunities such as “new infrastructure.” In addition, the government and e-commerce platforms should jointly build a live broadcast platform, orderly guide more market players to participate in the construction, reasonably reduce the platform costs or open up special channels to help farmers, and enhance the enthusiasm of farmers to participate, so as to realize the value co-creation of live broadcast e-commerce to help rural revitalization strategic practice.

RETRACTED

Figure 7 shows the satisfaction with the diversified system of rural industrial integration Internet platform between different cities driven by e-commerce. It can be seen that Beijing and Shanghai residents are the most satisfied with the rural industrial integration Internet platform, followed by Chongqing and finally Tianjin. In addition, the satisfaction of urban residents in Beijing is relatively stable, with little fluctuation, while the satisfaction of the other three cities is large and has no specific rules. This shows that Beijing has a better Internet application foundation, which can attract different e-commerce companies to invest in production, so as to promote the upgrading and development of rural industries and achieve the goal of rural revitalization.  Figure 8 shows the average satisfaction with the diversified system of rural industrial integration Internet platform between different cities driven by e-commerce. We can conclude that the average satisfaction of Beijing and Shanghai is higher than 80%, that of Chongqing is as high as 77.5%, and that of Tianjin is the lowest, only 72.5%. In short, to improve the satisfaction of residents in different cities, we should formulate corresponding measures to change the rural industry according to the characteristics of each city and local conditions. At the same time, it should be closely combined with the Internet to promote the transformation of rural industry and realize the digital and networked development.

## 4. Conclusion

The rapid development of e-commerce has promoted the wide application of the Internet, and the development of rural industries is closely related to the Internet. Driven by e-commerce, this paper integrates rural industry and Internet, studies the functional principle of rural industry integration Internet in detail, and establishes the right application platform. Then, the application of rural industry integration Internet platform to different cities reveals the dilemma of rural revitalization and puts forward optimization ways, which is of great significance, provides ideas and points out the direction for rural revitalization.

## Figures and Tables

**Figure 1:** The commercial operation mode of rural industry integrating Internet driven by e-commerce.

**Figure 2:** Flow diagram of rural industrial integration Internet platform driven by e-commerce.

RETRACTED

**Figure 3:** The development of Internet platform for rural industrial integration between different cities driven by e-commerce.

**Figure 4:** The proportion rate of rural industry integration and Internet revitalization among different cities driven by e-commerce.

**Figure 5:** The educational background of talents in the Internet revitalization of rural industrial integration between different cities driven by e-commerce.

**Figure 6:** The fusion degree in the Internet revitalization of rural industrial integration between different cities driven by e-commerce.

**Figure 7:** Satisfaction with the diversified system of rural industrial integration Internet platform between different cities driven by e-commerce.

**Figure 8:** The average satisfaction with the diversified system of rural industrial integration Internet platform between different cities driven by e-commerce.

## Data Availability

The experimental data used to support the findings of this study are available from the corresponding author upon request.
